The article "FKBP14 overexpression contributes to osteosarcoma carcinogenesis and indicates poor survival outcome" was retracted in 2025. Reasons: results that could not be reproduced; plagiarized images; overlap with other authors' work.

# FKBP14 overexpression contributes to osteosarcoma carcinogenesis and indicates poor survival outcome

**DOI:** 10.18632/oncotarget.9524

**Published:** 2016-05-20

**Authors:** Zhongming Huang, Junhua Li, Shaohua Du, Yanghua Tang, Ligang Huang, Luwei Xiao, Peijian Tong

**Affiliations:** ^1^ Department of Orthopaedic Surgery, Affiliated Jiangnan Hospital of Zhejiang Chinese Medical University, Hangzhou 310053, China; ^2^ Department of Orthopaedic Surgery, Xiaoshan Chinese Medical Hospital of Zhejiang Chinese Medical University, Hangzhou 310006, China; ^3^ Zhejiang Chinese Medical University, Hangzhou 310053, China; ^4^ Institute of Orthopaedics and Traumatology of Zhejiang Province, Hangzhou 310053, China; ^5^ Department of Orthopedic Surgery, The Second Affiliated Hospital, School of Medicine, Zhejiang University, Hangzhou 310053, China; ^6^ Department of Orthopaedic Surgery, The First Affiliated Hospital of Zhejiang Chinese Medical University, Hangzhou 310053, China

**Keywords:** osteosarcoma, FKBP14, GSEA, proliferation, apoptosis

## Abstract

The FK506-binding protein 14 (FKBP14) is a subfamily of immunophilins, has been implicated in various biochemical processes. However, its effects on the primary malignant bone tumor, osteosarcoma, are unclear. Here, we reported that FKBP14 may be an oncogene as it overexpressed in osteosarcoma tissues and cell lines, and FKBP14 expression was correlated with metastases, recurrence, tumor maximum diameter and poor survival time. FKBP14 was associated with the biological pathways including cell cycle, apoptosis and metastasis. Furthermore, we detected FKBP14 knockdown induced cell cycle arrest, apoptosis, invasion and adhesion *in vitro*. FKBP14 knockdown decreased the protein levels of PCNA, CDK1 and CCNB1 that promotes cell cycle, increased Bax, caspase-3 and caspase-7 protein involved in promoting cell apoptosis, and increased KIF4A expression as well as decreased SMC4 and TMEM33 proteins that contribute to cell invasion and adhesion. In addition, FKBP14 knockdown also caused a significant inhibition in tumor growth *in vivo*. Then, we found that the protein RhoA was identified as a binding partner of FKBP14. Taken together, FKBP14 may act as an oncogene in osteosarcoma via suppressing apoptosis and promoting invasion and adhesion in osteosarcoma carcinogenesis. FKBP14 may be a prognostic factor and potential target for osteosarcoma treatment.

## INTRODUCTION

Osteosarcoma accounts for nearly 60% of malignant bone tumors in the children and young adults for whom the prognosis remains poor, especially when metastases are present at diagnosis [1]. It mainly reported that osteosarcoma has been considered as a kind of differentiation disease resulted from genetic and epigenetic changes which interfere in osteoblast differentiation from mesenchymal stem cells [2]. There is a high tendency to metastatic spread of patients with osteosarcoma in the present of metastases to lung, most commonly in the periphery of the lungs, at initial diagnosis which accounts for approximately 20%, in addition, 40% of patients with osteosarcoma occurs metastases at a later stage [3–5]. The clinical treatment for osteosarcoma is still difficult because of the high metastatic potential and resistance to conventional chemotherapy. Surgery combines with neoadjuvant and adjuvant chemotherapy have been regarded as a rapid treatment for osteosarcoma, thus, responsible for improved the survival rate of patients [6]. So far, many studies have focused on the osteosarcoma metastasis, but the explicit molecular mechanism of that is not fully understood.

The article "FKBP14 overexpression contributes to osteosarcoma carcinogenesis and indicates poor survival outcome" was retracted in 2025. Reasons: results that could not be reproduced; plagiarized images; overlap with other authors' work.

The changes of gene expression have been attracted attention from researchers, which are closely related to the tumourigenesis, progression and the osteosarcoma treatment efficacy. Notably, tumor suppressor genes including SASH1, P-Axl, and IFN-a were found to involve in the regulation of proliferation, cell cycle distribution, apoptosis and invasion ability [7–9]. Moreover, many studies presented before suggest that the biological implications triggered by these genes may be tightly associated with altering the specific signaling pathways and/or regulating the expression of proteins which are key mediators of cell growth, apoptosis, migration and invasion. For example, MACC1 was originally identified in primary and metastastic colon cancer, markedly higher expressed in osteosarcoma tissues and induced cell proliferation, attested cell cycle, evoked cell apoptosis in U-2OS cells via activation of Akt signaling pathway [10]. And, silencing of galectin-3 observed repression of osteosarcoma cell migration and invasion mainly through inhibition of FAK/Src/Lyn activation and β-catenin expression [11].

The FK506-binding proteins (FKBPs) are a subfamily of immunophilins and expressed in a broad range of organisms [12]. FKBP family members exhibit distinct subcellular localizations and bind specific protein targets, and implicated in various biological progresses, such as protein folding, trafficking and transcription [13]. FKBP38 trends to help anti-apoptotic proteins Bcl-2 and Bcl-X_L_ to localize at the mitochondrial membrane and protect cells against apoptosis [14]. FKBP51/heat shock protein 90 (HSP90) or FKBP52/HSP90 complexes are correlated with progesterone or glucocorticoid receptor and contribute to migration of the ternary complexes from the cytoplasm to the nucleus [15, 16]. Here, we investigated the function of one member of FKBP family, FKBP14, in osteosarcoma tumorigenesis. Researchers have shown previously that FKBP14 identification of a metastasis-associated gene in colon cancer [17] and mutations in FKBP14 results in Ehlers-Danlos syndrome which appearances of kyphoscoliosis, myopathy and hearing loss [18]. Despite the clear importance of the role of FKBPs in cancer and disease [19, 20], little is known about how FKBP14 involved in the tumorigenesis of osteosarcoma.

The article "FKBP14 overexpression contributes to osteosarcoma carcinogenesis and indicates poor survival outcome" was retracted in 2025. Reasons: results that could not be reproduced; plagiarized images; overlap with other authors' work.

In this study we show that FKBP14 overexpresses in osteosarcoma tissues and indicated a poor survival. Interestingly, FKBP14 knockdown remarkably inhibits U-2OS and MG63 cells proliferation, invasion, and adhesion and arrests cell cycle followed by cell apoptosis. Moreover, FKBP14 is correlated with cell cycle, apoptosis, invasion and metastasis biological pathways via regulating signaling pathway associated protein expressions. These findings support a potential role for FKBP14 as a tumor promoter and efficacy for a target for osteosarcoma treatment.

## RESULTS

### FKBP14 up-regulation in osteosarcoma tissues

To identify the genes differentially expressed in osteosarcoma, we compared the gene expression profiles of 83 patients' osteosarcoma tissues and 67 patients' bone cysts through microarray and immunohistochemistry analysis. Functional clustering analysis of the up-regulating genes exhibited a significant enrichment of genes associated with cell cycle, apoptosis and metastasis (data not shown). Among these genes, FKBP14 showed significant increase in mRNA level in the osteosarcoma tissues compared with the bone cysts of patients in Xiaoshan Chinese Medical Hospital (Figure 1A, *P* < 0.01). Moreover, immunohistochemical examination of FKBP14 was showed that 83 osteosarcoma tissues showed higher level of FKBP14 expression, 51 with lower expression and 16 tissues with no expression of FKBP14 (Figure 1B). These data suggest that FKBP14 may be an oncogene in osteosarcoma.

**Figure 1:** FKBP14 up-regulation in osteosarcoma tissues and regulates biological pathways (**A**) Microarray analysis of FKBP14 expression in bone cysts and osteosarcoma in Xiaoshan Chinese Medical Hospital; (**B**) Representative immunohistochemical staining for FKBP14 in osteosarcoma tissues. Survival analysis showed that FKBP14-lower expression tumors have a favorable prognosis compared with FKBP14-higher expression tumors; (**C**) The overall survival time of 150 osteosarcoma patients from Xiaoshan Chinese Medical Hospital; (**D**) The metastase-free survival time of 81 osteosarcoma patients from Xiaoshan Chinese Medical Hospital; (**E**) The overall survival time of 37 osteosarcoma patients from GSE39055 database. GSEA compared FKBP14 higher expression group (red) against FKBP14 lower expression group (blue) of osteosarcoma patients in the E-MEXP-3628 dataset. Enrichment plots are shown for a set of activated genes related to (**F**) cell cycle, (**G**) apoptosis and (**H**) metastasis. **P < 0.01 compared with bone cysts.

The article "FKBP14 overexpression contributes to osteosarcoma carcinogenesis and indicates poor survival outcome" was retracted in 2025. Reasons: results that could not be reproduced; plagiarized images; overlap with other authors' work.

### FKBP14 expression associates with clinical characteristics and regulates biological pathways in osteosarcoma pathogenesis

To examine the association of FKBP14 expression with clinicopathologic variables in osteosarcoma patients, we collected 150 osteosarcoma patient samples. The osteosarcoma patients were divided into two groups according to the mean level of FKBP14. The clinical and histopathological details of the 150 cases were listed in Table 1. FKBP14 expression was positive correlated with the metastases, recurrence and tumor maximum diameter. Next, we explored the correlation of FKBP14 expression with the poor prognosis. As known in Figure 1C (*P* = 0.0001) and D (*P* = 0.0353), Kaplan-Meier analysis showed that the overall survival time and metastasis-free survival time of FKBP14-lower-expressed was notably higher than that of FKBP14-higher-expressed patients. We also analyzed data of osteosarcoma patients from GEO dataset (Access id: GSE39055) that the survival time was significantly shorter of patients with FKBP14-higher-expressed tumors than that of patients with FKBP14-lower-expressed tumors (Figure 1E, *P* = 0.025). These results all support our findings that FKBP14 could represent a new prognostic factor in osteosarcoma patients.

**Table 1:** Relationship between FKBP14 and clinical characteristics of osteosarcoma patients

Factor	Characteristic	FKBP14 expression (N)		*P*-values
		Lower	Higher	
Gender	Male	33	41	1.0000
	Female	34	42	
Age (years)	< 18	40	51	0.8675
	> = 18	27	32	
Enneking's stage	I	10	7	0.6529
	IIA	20	25	
	IIB	31	43	
	III	6	8	
Tumor location	Femur	37	39	0.8175
	Fibula	5	10	
	Tibia	9	13	
	Humerus	7	8	
	Others	9	13	
Metastases	Lung	16	31	0.0356*
	Other	7	15	
	No	44	37	
Recurrence	Yes	15	39	0.0018**
	No	52	44	
Tumor maximum diameter (cm)		4.36 ± 0.21	5.81 ± 0.38	0.0019^##^

* *P* < 0.05,

** *P* < 0.01, Chi-square test.

## *P* < 0.01, student's *t* test.

To elucidate how FKBP14 promotes osteosarcoma pathogenesis, GSEA analysis was performed to gain further insight into the biological pathways in E-MEXP-3628 dataset. GSEA is used to detect coordinated differences in expression of predefined sets of functionally related genes. Among all the predefined gene sets, the cell cycle, apoptosis and metastasis pathways were identified with the strongest association with FKBP14 expression, which showed that the gene signatures of cell cycle, apoptosis and metastasis were correlated with the patients with FKBP14-higher-expressed compared with FKBP14-lower-expressed (Figure 1F–1H, *P* < 0.05).

The article "FKBP14 overexpression contributes to osteosarcoma carcinogenesis and indicates poor survival outcome" was retracted in 2025. Reasons: results that could not be reproduced; plagiarized images; overlap with other authors' work.

### Different expression and knockdown of FKBP14 in osteosarcoma cell lines

To validate the GSEA analysis of FKBP14, we examined the expression of FKBP14 in five different osteosarcoma cell lines, including HOS, 143B, U-2OS, SaoS2 and MG63 cells, and in normal chondrocyte. Real-time PCR and Western blot analysis showed that the expression of FKBP14 was significantly higher in U-2OS and MG63 cells compared with the normal chondrocyte, while FKBP14 was expressed in lower level in 143B cells (Figure 2A and 2B).

**Figure 2:** FKBP14 expression in osteosarcoma cell lines FKBP14 expression was measured by (**A**) Real-time PCR and (**B**) Western blot; Knockdown of FKBP14 by shRNA showed notably expression inhibited in (**C**) mRNA and (**D**) protein levels in U-2OS and MG63 cells; Overexpression of FKBP14 showed notably expression increased in (**E**) mRNA and (**F**) protein levels in 143B cells. **P < 0.01 compared with NC group. NC: negative control.

In order to knockdown FKBP14, we also introduced pLVX-AcGFP-C1 lentiviral vector expressing FKBP14 shRNA (sh-FKBP14) into U-2OS and MG63 cells. The efficacy of FKBP14 knockdown was examined by Real-time PCR and Western blotting. Meanwhile, a lentiviral vector expressing scramble shRNA was used as a negative control (NC). As shown in Figure 2C (*P* < 0.01), the mRNA levels of FKBP14 were decreased 81.6% and 63.2% in U-2OS and MG63 cells after infected with sh- FKBP14, respectively. 79.1% and 77.8% reduction were also found in protein level of U-2OS and MG63 cells after infected with sh-FKBP14 (Figure 2D, *P* < 0.01). Moreover, pLVX-AcGFP-C1-FKBP14 (FKBP14) expressing vector was stably infected into 143B cells (Figure 2E and 2F, *P* < 0.01). The mRNA levels of FKBP14 were increased by 1.62-fold in 143B cells after infected with pLVX-AcGFP-C1-FKBP14 compared with black pLVX-AcGFP-C1 infected 143B cells (NC).

### FKBP14 knockdown inhibits proliferation *in vitro* and *in vivo*

Next, we determined whether FKBP14 knockdown affects the osteosarcoma cell proliferation at progressive stages of tumorigenesis. Towards this end, cells were infected with sh-FKBP14 and cellular proliferation was determined using CCK-8 assay. We noted that FKBP14 knockdown remarkably inhibited the proliferation of U-2OS and MG63 cells after 48 h and 72 h (Figure 3A and 3B, *P* < 0.01). While, overexpression of FKBP14 in 143B cells increased cell proliferation compared with NC group (Figure 3C, *P* < 0.01).

The article "FKBP14 overexpression contributes to osteosarcoma carcinogenesis and indicates poor survival outcome" was retracted in 2025. Reasons: results that could not be reproduced; plagiarized images; overlap with other authors' work.

**Figure 3:** FKBP14 knockdown inhibits cell proliferation *in vitro* and *in vivo* (**A**, **B**) FKBP14 knockdown inhibits U-2OS and MG63 cells proliferation *in vitro*; (**C**) FKBP14 overexpression promotes 143B cells proliferation *in vitro*; (**D**) FKBP14 expression was measured by Western blot; (**E**) FKBP14 knockdown inhibits tumor growth in nude mice xenograft model *in vivo*; (**F**) Tumor volume and (**G**) weight were also measured after FKBP14 knockdown. **P < 0.01 compared with NC group. NC: negative control.

Next, we determined the effect of FKBP14 knockdown on the tumor growth *in vivo*. MG63 cells injected with NC or FKBP14-shRNA were subcutaneously injected in athymic nude mice respectively, and tumor volumes were measured for 36 days. The significantly decreased expression of FKBP14 was shown in Figure 3D. As shown in Figure 3E, FKBP14 down-regulated tumors grew slower in mice compared with the NC tumors in mice. After 36 days, tumor volume as well as tumor weight in FKBP14 down-regulated mice was also examined, which observed that the tumor volume and weight in FKBP14 down-regulated mice were significant decrease compared with those in NC mice (Figure 3E and 3F, *P* < 0.01). These data suggest that inhibition of FKBP14 in osteosarcoma reduce tumor growth in nude mice.

### FKBP14 knockdown arrests cell cycle at G0/G1 phase *in vitro*

To dissect the mechanism for the anti-proliferative effects of FKBP14 knockdown, we considered whether the proliferation inhibitory effects of FKBP14 knockdown are associated with specific changes in cell cycle progression. U-2OS and MG63 cells were infected with sh-FKBP14 for 48 h and harvested for flow cytometry analysis by PI staining. As shown in Figure 4A, FKBP14 knockdown of U-2OS cells caused an increase in the number of cells in the G0/G1 phase of the cell cycle, providing evidence of G0/G1 arrest. At the same time, the G0/G1 population increased from 46.7% in the NC group to 59.9% in the U-2OS cells and increased from 52.1% in the NC group to 65.7% in the MG63 cells infected with sh-FKBP14, respectively, and with a concomitant decrease in the percentage of S phase cells (Figure 4B, *P* < 0.01). Interestingly, we observed a dramatic decrease in proliferating cell nuclear antigen (PCNA), cyclin-dependent kinases 1 (CDK1) and cyclin B1 (CCNB1) protein levels upon down-regulation of FKBP14 in both U-2OS and MG63 cells (Figure 4C and 4D, *P* < 0.01). These data demonstrate that FKBP14 knockdown resulted in the G0/G1 phase arrest in both U-2OS and MG63 cells.

**Figure 4:** FKBP14 knockdown induces cell cycle arrest Cell cycle arrested at G1 phase after FKBP14 knockdown in (**A**) U-2OS and (**B**) MG63 cells assessed by flow cytometry; Expressions of cell cycle markers (PCNA, CDK1 and CCNB1) were significantly down-regulated after FKBP14 knockdown in (**C**) U-2OS and (**D**) MG63 cells. **P < 0.01 compared with NC group. NC: negative control.

The article "FKBP14 overexpression contributes to osteosarcoma carcinogenesis and indicates poor survival outcome" was retracted in 2025. Reasons: results that could not be reproduced; plagiarized images; overlap with other authors' work.

### FKBP14 knockdown induces cell apoptosis *in vitro*

To investigate and confirm the appearance of cell apoptosis, we evaluated the apoptotic function of FKBP14 in U-2OS and MG63 cells by Annexin V-FITC/PI staining assay. As shown in Figure 5A and 5B, flow cytometry analysis revealed that knockdown of FKBP14 in U-2OS and MG63 cells significantly increased cell apoptosis by 6.6-fold and 7.7-fold compared with the corresponding NC groups. While, overexpression of FKBP14 in 143B cells reduced cell apoptosis compared with NC (Figure 5C, *P* < 0.01). Down-regulation of FKBP14 in both U-2OS and MG63 cells resulted in a significantly increase in Bax, caspase-3 and caspase-7 protein levels (Figure 5D and 5E, *P* < 0.01). While, overexpression of FKBP14 in 143B cells decreased the expression of Bax, caspase-3 and caspase-7 (Figure 5F, *P* < 0.01). These results indicate that the anti-proliferation function of FKBP14 knockdown was most likely mediated by inhibiting G1/S cell cycle transition and inducing apoptosis.

**Figure 5:** FKBP14 knockdown induces cell apoptosis Cell apoptosis was significantly increased after FKBP14 knockdown in (**A**) U-2OS and (**B**) MG63 cells and decreased in (**C**) 143B cells with FKBP14 overexpression, assessed by flow cytometry; Expressions of apoptosis markers (Bax, caspase-3 and caspase-7) were significantly up-regulated after FKBP14 knockdown in (**D**) U-2OS and (**E**) MG63 cells and were down-regulated after FKBP14 overexpression in (**F**) 143B cells. **P < 0.01 compared with NC group. NC: negative control.

### FKBP14 knockdown inhibits cell invasion and adhesion *in vitro*

We wonder whether FKBP14 regulated metastasis of osteosarcoma cells. To investigate the invasion-promoting function of FKBP14 in osteosarcoma cells, the invasion capacity of U-2OS and MG63 cells were evaluated by transwell assay. As shown in Figure 6A (*P* < 0.01), sh-FKBP14 infected into U-2OS and MG63 cells significantly reduced the invasive capacity by 47.5% and 52.5% compared with the corresponding NC groups. Furthermore, we also detect the adhesive capacity of U-2OS and MG63 cells with sh-FKBP14 treatment. The results observed that FKBP14 knockdown notably repressed the U-2OS and MG63 cells adhesive ability by 54.1% and 59.8% compared with the corresponding NC groups (Figure 6B, *P* < 0.01). However, overexpression of FKBP14 in 143B cells promoted cell invasion and adhesion compared with NC (Figure 6A and 6B, *P* < 0.01). Additionally, our results showed that the expressions of structural maintenance of chromosomes protein 4 (SMC4) and transmembrane protein 33 (TMEM33) were remarkably decreased in both U-2OS and MG63 cells treated with sh-FKBP14, while the expression of kinesin family member 4A (KIF4A) was increased (Figure 7A and 7B, *P* < 0.01). Other invasion and adhesion factors were also measured in 143B cells and we found that Twist1, Snail1, Snail2, matrix metalloprotein 2 (MMP2) and MMP9 were significantly increased in 143B cells with FKBP14 overexpression compared with NC, with E-cadherin exception (Figure 7C, *P* < 0.01). Taken together, these results suggest that FKBP14 knockdown suppresses the invasion and adhesion of osteosarcoma cells.

The article "FKBP14 overexpression contributes to osteosarcoma carcinogenesis and indicates poor survival outcome" was retracted in 2025. Reasons: results that could not be reproduced; plagiarized images; overlap with other authors' work.

**Figure 6:** FKBP14 knockdown inhibits cell invasion and adhesion (**A**) Cell invasion and (**B**) adhesion were significantly inhibited after FKBP14 knockdown in U-2OS and MG63 cells and were increased in 143B cells, respectively. **P < 0.01 compared with NC group. NC: negative control.

**Figure 7:** Effect of FKBP14 knockdown on the expression of proteins correlated with invasion and adhesion Expressions of invasion and adhesion markers were significantly up-regulated (KIF4A) or down-regulated (SMC4 and TMEM33) after FKBP14 knockdown in (**A**) U-2OS and (**B**) MG63 cells; (**C**) Expressions of other invasion and adhesion markers were significantly down-regulated (E-cadherin) or up-regulated (Twist1, Snail1, Snail2, MMP2 and MMP9) after FKBP14 overexpression in 143B cells. **P < 0.01 compared with NC group. NC: negative control.

### Association of FKBP14 with RhoA

To elucidate the underlying mechanisms by which FKBP14 exerts its function in osteosarcoma pathogenesis, we identified protein candidates that functionally associated with FKBP14. As shown in Figure 8A and 8B, we explored the nature of the interaction between FKBP14 and RhoA by using Co-immunoprecipitiation in both U-2OS and MG63 cells. The result obtained from the Co-immunoprecipitiation experiments indicated that RhoA directly interacts with FKBP14.

**Figure 8:** FKBP14 binds to RhoA *in vitro* Co-immunoprecipitation showed that FKBP14 interacts with RhoA in the cell lines (**A**) U-2OS and (**B**) MG63 cells.

## DISCUSSION

FKBP14 expression levels in osteosarcoma patients were evaluated. Previous studies reported that FKBP14 is frequently upregulated in a variety of human malignancies [21]. In the current study, FKBP14 mRNA expression levels were higher in osteosarcoma patients compared with bone cysts patients, and this difference was significant. Patients with higher-expressed FKBP14 had significantly shorter survival periods than those with lower-expressed FKBP14. These findings of the present study indicate that FKBP14 expression induced by osteosarcoma can be considered as a diagnostic biomarker. GSEA analysis demonstrated that the cell cycle, apoptosis and metastasis biological pathways were significantly enriched in response to FKBP14 alternation in osteosarcoma patients. The bioinformatic analysis was further validated in the subsequently performed *in vitro* and *in vivo* experiments.

The article "FKBP14 overexpression contributes to osteosarcoma carcinogenesis and indicates poor survival outcome" was retracted in 2025. Reasons: results that could not be reproduced; plagiarized images; overlap with other authors' work.

In cultured osteosarcoma cell lines, we found that U-2OS and MG63 cells presented a highly expression of FKBP14 and 143B cells with a low levels of FKBP14 expression in comparison with other osteosarcoma cells, thus these three cells were used for our following experiments to investigate the roles for FKBP14 in osteosarcoma via RNA interfering or overexpression. The proliferation inhibitory effects of FKBP14 *in vitro* and *in vivo* prompted us to investigate whether this is associated with regulations of the proteins of biological pathways. FKBP14 knockdown tremendously reduced cell cycle associated protein expression, including PCNA, CDK1 and CCNB1. PCNA is manly expressed during the G1, S and G2 phases of the cell cycle [22]. This is in agreement with others findings showing that reduced expression of PCNA accompanied with G0/G1 phase arrest of hematopoietic progenitor cells [23]. The abundance of CCNB1 mRNA and protein increased normally from G1 to G2 phase and the phosphorylation of CDK1 was decreased in hepatocytes as the cells proceeded through G2/M phase [24]. The reduced expression of CCNB1 and CDK1 is mediated in part by p53-dependent repression of the CCNB1 and CDK1 promoters [25].

Whereas apoptosis involves in an energy-dependent mechanism where cells participate in their own destruction resulted from necrosis [26]. Importantly, the effect of FKBP14 knockdown to induce apoptosis in U-2OS and MG63 cells was contributed to an increase in the expression of Bax followed by the expression of caspase-3 and caspase-7. Loss of the Bax protein function may play an important role in the pathogenesis of many types of cancer [27, 28]. The inhibition of apoptosis appears to occur through the down-regulation of Bax and caspase-3 in osteosarcoma cells, which thereby prevent apoptotic cascades [29]. It is worth mentioning that FKBP14 knockdown induced up-regulation of Bax, caspase-3 and caspase-7 level in U-2OS and MG63 cells providing further support to the hypothesis that down-regulation of FKBP14 is more likely to elicit its apoptotic and therapeutic effects on osteosarcoma tumorigenesis.

Invasion through the extracellular host matrix and adherence and survival in the target organ site were critical steps to complete the metastasis [30]. Our data showed that the effect of FKBP14 knockdown on invasion and adhesion was dependent of regulation of related proteins, such as KIF4A, SMC4 and TMEM33. In an early study, loss of KIF4A might lead to carcinogenesis via inducing proliferation as well as growth of tumor *in vivo* [31]. In contrast, KIF4A positive tumors revealed an enhanced the cellular invasion *in vitro* assay, suggesting KIF4A is associated with a highly invasion phenotype of mammalian cells [32]. Therefore, further works need to better understand the complex roles of KIF4A plays in development and progresses of cancer. Zhou et al. reported that the expression of SMC4 is correlated with vascular invasion of primary liver cancers [33]. In melanoma, TMEM33 was found positively correlated with neutral endopeptidase (NEP), which has been reported in metastatic carcinomas and regulated genes of focal adhesion in melanoma [34]. Other markers were also measured in 143B cells with FKBP14 overexpressing vector infection. We found that Twist1, Snail1, Snail2, MMP2 and MMP9 were significantly increased, with E-cadherin exception. Consistent with the previous studies, transfection with Twist1 shRNA dramatically inhibited cell migration in osteosarcoma [35]. Overexpression of Snai1 in osteosarcoma is associated with tumor progression, possibly through the suppression of E-cadherin [36]. Snail2 was expressed in high-grade cranial bone osteosarcomas correlated with osteosarcoma metastasis and may be a useful prognostic marker for this disease [37]. Moreover, disulfiram, a chelator of heavy metals and an inhibitor of aldehyde dehydrogenase, suppressed MMP2 and MMP9 activity and expression, producing an almost complete growth and invasion inhibition of osteosarcomas cells, suggesting an important role of MMP2 and MMP9 in tumor growth and metastasis [38].

The article "FKBP14 overexpression contributes to osteosarcoma carcinogenesis and indicates poor survival outcome" was retracted in 2025. Reasons: results that could not be reproduced; plagiarized images; overlap with other authors' work.

Recent studies have demonstrated the functional interaction of FKBP14 with Psn protein in the endoplasmic reticulum, which is essential for effective Notch signal transduction [39]. In this study, we revealed that FKBP14 directly bound to RhoA in both U-2OS and MG63 cells, suggesting that implicate signaling through RhoA pathway as a critical downstream mechanism by which FKBP14 may regulate changes in the cell proliferation, cell cycle, apoptosis and invasion. One of the important Wnt signaling mediators, the small GTPase RhoA, was shown to play an oncogenic role in osteosarcoma [40]. RhoA inactivation induced osteosarcoma cell apoptosis by inhibiting p42/p44-MAPKs-Bcl-2 signaling [41]. Inhibition of RhoA reduces osteosarcoma cell invasion and MMP2 activity [42].

In conclusion, the results presented in this study provided additional insight into the mechanisms of osteosarcoma tumorigensis. Our study provides for the first time that FKBP14 played an important role in proliferation, cell cycle, apoptosis, invasion and adhesion in osteosarcoma cells. As FKBP14 expression level associated with patients' survival time, it might be a useful prognostic factor for osteosarcoma.

## MATERIALS AND METHODS

### Patient specimens

Osteosarcoma tissues and bone cyst specimens were obtained from patients who underwent surgery at Xiaoshan Chinese Medical Hospital from Feb 2000 to May 2010. The study protocol was approved by the ethics committee of Xiaoshan Chinese Medical Hospital. Written informed consents were obtained from all participants in this study. All the research was carried out in accordance with the provisions of the Helsinki Declaration of 1975.

### Bioinformatics analysis

Survival rate data was downloaded from the NCBIs Gene Expression Omnibus (GEO, http://www.ncbi.nlm.nih.gov/geo/) and are accessible through GEO Series accession number GSE39055. To gain further insight into the biological pathways involved in osteosarcoma pathogenesis through FKBP14 pathway, a gene set enrichment analysis (GSEA) was performed [43]. The GSEA data was obtained from the E-MEXP-3628 database.

### Cell culture

Osteosarcoma cell lines (HOS, 143B, U-2OS, SaoS2 and MG63) and normal chondrocyte were purchased from the Academia Sinica Cell Bank (Shanghai, China). HOS, 143B and MG63 cells were cultured in DMEM (Life Technologies, Carlsbad, CA, USA) supplemented with 10% fetal bovine serum (FBS, Biowest) and 1% penicillin-streptomycin solution (Gibco). SaoS2 cells were grown in DMEM with 15% FBS and 1% penicillin-streptomycin solution. U-2OS cells were grown in RPMI 1640 (Biowest) with 10% FBS and 1% penicillin-streptomycin solution. Cells were cultured at 37°C in an atmosphere of 5% CO_2_.

### Lentivirus transduction

The FKBP14 shRNA or cloning sequence was cloned into the pLVX-AcGFP-C1 lentiviral vector. A scramble shRNA cloned into pLVX-AcGFP-C1 lentiviral vector and black pLVX-AcGFP-C1 lentiviral vector were used as negative control (NC), respectively. The constructs were then transducted into HEK 293T cells with lentiviral packaging vectors by using lipofectamine 2000 (Invitrogen) according to the manufacture's instruction. After 48 h transduction, lentivirus was collected and infected U-2OS and MG63 or 143B cells.

### Cell proliferation assay

The proliferation effects of the FKBP14 on the cells were determined by Cell Count Kit-8 (CCK-8, Dojindo, Rockville, MD, USA) assay. Briefly, control and infected U-2OS and MG63 or 143B cells were plated in 96-well plates at an initial density of 1 × 10^4^ cells per well. CCK- 8 solution (100 μL/well) was added to the cells at 0 h, 24 h, 48 h and 72 h. Then cells were cultured at 37°C in an atmosphere of 5% CO_2_ for 1 h. The reaction product was quantified by measured the absorbance at wavelength 450 nm using the plate reader Multiskan EX (Thermo Fisher Scientific Inc., Waltham, MA, USA).

The article "FKBP14 overexpression contributes to osteosarcoma carcinogenesis and indicates poor survival outcome" was retracted in 2025. Reasons: results that could not be reproduced; plagiarized images; overlap with other authors' work.

### Cell cycle assay

The percentages of cells in the different phases of cell cycle were evaluated by determining the DNA content after propidium iodide (PI) staining (BiovisionInc, Mountain View, CA, USA). Briefly, control and infected U-2OS and MG63 cells were plated in 6-well plates at an initial density of 3 × 10^5^ cells per well. Then Cells were fixed in cold ethanol for 24 h at 4°C and then incubated with propidium iodide (PI, 50 μg/mL) for 10 min before flow cytometry analysis (BD Biosciences, San Diego, CA).

### Cell apoptosis assay

An annexin-V fluorescein isothiocyanate (FITC)/PI double stain assay (Biovision Inc, Mountain View, CA) were performed following the manufacturer's protocol. Briefly, control and infected U-2OS and MG63 or 143B (1 × 10^5^) cells were resuspended with 195 μL Annexin V and 5 μL PI and incubated for 5 min in the dark at room temperature before flow cytometry analysis.

### Cell invasion and adhesion assay

Invasion assays were performed using Transwell chamber (Greiner Bio-One, Frickenhausen, Germany) coated with Matrigel (BD, San Diego, CA, USA) as described in the manufacturer's protocol. Briefly, control and infected U-2OS and MG63 or 143B (3 × 10^5^) cells were plated in the top chamber of the insert precoated with Matrigel. For adhesion assay, 1 × 10^5^ cells/well were seeded on fibronectin-coated 12-plate microplate and incubated for 1 h at 37°C in an atmosphere of 5% CO_2_. The cells were fixed with 4% paraformaldehyde (Gibco) for 10 min and stained with Giemsa (Gibco) for 30 min. Cells were photographed and counted under microscopy in random 10 fields with magnification of ×200.

### RNA extraction and Real-time PCR

Total RNAs were extracted from osteosarcoma tissues and bone cyst or osteosarcoma cells with TRIZOL reagent (Life Technologies) according to the manufacturer's protocol. Real-time PCR was performed using SYBR Green qPCR kit (Finnzymes Oy, Espoo, Finland). GAPDH level was used as internal control and expression changes were calculated using the 2^−ΔCt^ method [44]. The primers sequences (sense/antisense) used were list as follows: FKBP14, 5′-TGAAGGACAGCACCAATAG-3′ and 5′-GCACATTT ACCACCAACTC-3′; GAPDH: 5′-CACCCACTCCTCCA CCTTTG-3′ and 5′-CCACCACCCTGTTGCTGTAG-3′.

### Western blot

Total proteins were isolated from control and infected U-2OS and MG63 or 143B cells, and were subjected to 12% SDS-PAGE and electrophoretically transferred onto a nitrocellulose sheet. Membranes were first incubated with antibody against FKBP14, PCNA, CDK1, CCNB1, Bax, caspase-3, caspase-7, KIF4A, SMC4, TMEM33, Twist1, Snail1/2, MMP2/9 and E-cadherin, then with anti-GAPDH antibody as an internal control. Antibodies used in this study were purchased from Abcam (Cambridge, MA, USA), unless otherwise specified: Bax and TMEM33 (Santa Cruz Biotechnology, Santa Cruz, CA, USA) and GAPDH (CST Biotech, Danvers, MA, USA).

The article "FKBP14 overexpression contributes to osteosarcoma carcinogenesis and indicates poor survival outcome" was retracted in 2025. Reasons: results that could not be reproduced; plagiarized images; overlap with other authors' work.

### Co-immunoprecipitation (Co-IP)

Co-immunoprecipitation was performed as described previously [45]. Both the input and IP samples were analyzed by Western blot using various antibodies at the following dilutions: FKBP14 antibody (1:1000), RhoA antibody (1:1000), Flag-tag antibody (1:1000), HA-tag antibody (1:1000) and normal rabbit/mouse IgG (Cell Signaling Technology).

### Immunohistochemical analysis

Immunohistochemistry (IHC) for the detection of FKBP14 was performed on sections of patients' tumor tissues. And immunohistochemistry were performed as previously described. The results of IHC staining were evaluated independently by two trained pathologists without knowledge of clinical data. The specimens were graded into three groups according to the extent of positivity as follows: Negative: no positive stain; Low: < 25% of the tumor cells showed positive stain; high: > 25% of tumor cells showed positive stain. The slides were reexamined by the pathologists together and an agreement reached regarding the final evaluation.

### *In vivo* experiments

In order to clarify the role of FKBP14 *in vivo*, 6-week-old male athymic nude mice were used in this study. 12 male athymic nude mice were randomly divided into 2 groups (6 mice per group). MG63 cells (2 × 10^6^) with negative control or FKBP14-shRNA were injected subcutaneously into the right flank of these mice to establish the osteosarcoma xenograft model. At 5 weeks after injection, the mice were euthanized and the tumors were weighted. All the experiments were approved by Hangzhou Medical Experimental Animal Care Commission.

### Statistical analysis

The data was presented as the mean value ± s.d. The paired, two-tailed Student's *t*-test was used to analyze the significance of difference between groups. The Chi-square tests were used to compare the clinicopathologic characteristics of tumors (and patients) with high and low FKBP14 expression. Overall survival in relation to FKBP14 expression was evaluated by the Kaplan-Meyer survival curve and the log-rank nonparametric test. Differences were considered significant with a value of *P* < 0.05.
